RETRACTED

# Prediction Model of Hot Metal Silicon Content Based on Improved GA-BPNN

**DOI:** 10.1155/2021/1767308

**Published:** 2021-08-17

**Authors:** Zeqian Cui, Yang Han, Chaomeng Lu, Yafeng Wu, Mansheng Chu

**Affiliations:** ^1^College of Metallurgy and Energy, North China University of Science and Technology, Tangshan, Hebei, China; ^2^Tangshan Key Laboratory of Engineering Computing, College of Science, North China University of Science and Technology, Tangshan, China; ^3^College of Science, North China University of Science and Technology, Tangshan, Hebei, China; ^4^College of Artificial Intelligence, North China University of Science and Technology, Tangshan, Hebei, China; ^5^School of Metallurgy, Northeastern University, Shenyang, Liaoning, China

## Abstract

The inconsistency of the detection period of blast furnace data and the large time delay of key parameters make the prediction of the hot metal silicon content face huge challenges. Aiming at the problem that the hot metal silicon content is not consistent with the detection period of time series of multiple control parameters, the cubic spline interpolation fitting model was used to realize the data integration of multiple detection periods. The large time delay of the blast furnace iron making process was analyzed. Moreover, Spearman analysis was combined with the weighted moving average method to optimize the data set of silicon content prediction. Aiming at the problem of low prediction accuracy of the ordinary neural network model, genetic algorithm was used to optimize parameters on the BP neural network model to improve the convergence speed of the model to achieve global optimization. Combined with the autocorrelation analysis of the hot metal silicon content, a modified model for the prediction of hot metal silicon content based on error analysis was proposed to further improve the accuracy of the prediction. The model comprehensively considers problems such as data detection inconsistency, large time delay, and inaccuracy of prediction results. Its average absolute error is 0.05009, which can be used in actual production.

## 1. Introduction

In the steel production process, the blast furnace provides high-quality hot metal for steelmaking through complicated processes such as discrete addition, continuous smelting, and discrete output. The control parameters of the smelting process have more than 100 and have the characteristics of high nonlinearity, randomness, and large time lag, so controlling the stable state of the furnace temperature is one of the keys to ensure the smooth progress of blast furnace ironmaking [1–4]. Due to the complex internal environment of the blast furnace and the interference of various physical and chemical factors, it is difficult to accurately monitor the furnace temperature. Production practice shows that the hot metal silicon content has a strong correlation with the temperature of the blast furnace, and it can be used to indirectly reflect the temperature change in the furnace [5–8].

RETRACTED

In recent years, many researchers have researched the prediction of hot metal silicon content. Liu et al. compared the prediction effects of the three models, including random forest, AdaBoost, and decision tree. They found that the AdaBoost model had better predictive validity, but the model is too sensitive to abnormal samples [9]. Huang et al. improved the accuracy of prediction of hot metal silicon content by combining principal component analysis with extreme learning machine and optimizing the weight and threshold using particle swarm optimization algorithm. But they did not consider the large time lag of the smelting process [10]. Li et al. derived the calculation formula of hot metal silicon content through the analysis of the data of charge, blast furnace gas and slag iron temperature, and compared it with the actual results. However, the intelligent application of the model is less [11]. Although Li et al. predicted the hot metal silicon content by the LSTM-RNN model and compared it with PLS and RNN models, data processing and analysis of this model were rarely carried out [12]. With the advent of the era of big data, data-driven methods have attracted wide attention. Affected by factors such as the accuracy of the existing detection technology and the complex operating conditions of the blast furnace, the use of data-driven methods requires consideration of the integrity and volatility, as well as the time lag characteristics of the data [13–16]. Therefore, it is very important to choose a suitable mathematical model to mine the useful information in the data.

For the above reasons, a back-propagation neural network optimized by genetic algorithm (GA-BPNN) hot metal silicon content error correction prediction model based on data optimization is proposed. In order to achieve accurate prediction of the hot metal silicon content in the complex environment of the blast furnace, multiple control parameters, such as coal injection rate, hot air pressure, hot air temperature, air permeability, and oxygen-enriched flow rate, should be fully used as inputs [17, 18]. However, multiple data input is accompanied by inconsistent data detection periods and large time lags in key parameters, so it is necessary to optimize and integrate the data [19]. That is, through the analysis of the trend and correlation of the data, the data set that is helpful for the subsequent prediction of the silicon content of the molten iron is extracted, which is data optimization. The nonlinear and high-dimensional characteristics of blast furnace data [20] require the model to have good nonlinear mapping capabilities and adaptive capabilities. The accuracy of the prediction model of hot metal silicon content can be further improved by combining with the characteristics of strong time series of the hot metal silicon content [21].

RETRACTED

## 2. The Proposed Model

### 2.1. Data PreProcessing

Outlier elimination: the 3*σ* criterion is used to eliminate outliers in the blast furnace sample set. Suppose the sample set is *X* = {*x*_1_,…, *x*_*n*_}, when the absolute value of the difference between the value *x*_*i*_ and the average value $\bar{x}$ is greater than 3*σ*, it will be regarded as an outlier and eliminated [22, 23]. The calculation formula of *σ* is

(1) $$\begin{array}{c} \sigma =\;\sqrt{\overset{n}{\underset{i=1}{\sum }}\frac{e_{i}^{2}}{\left(n-1\right)}}=\;\sqrt{\overset{n}{\underset{i=1}{\sum }}\frac{{\left(x_{i}-\bar{x}\right)}^{2}}{\left(n-1\right)}}. \end{array}$$

Here, $\bar{x}$ is the average value.

The data distribution of the silicon content of the molten iron is shown by the box plot method, as shown in Figure 1. It can be seen that the silicon content of molten iron is mostly concentrated around 0.5.

Normalization: in the process of blast furnace ironmaking, the data dimensions are quite different. For example, the range of blast furnace permeability index is between [50, 100], and the range of cold air flow parameters is [1800, 2300]. It is obviously unreasonable to apply them directly to the prediction of the hot metal silicon content, which makes a wide range of data have a great influence on the prediction result. For the accuracy of subsequent model predictions, the data normalization method is used to control the range of control parameters such as coal injection amount and wind pressure between [0, 1]. The calculation formula is

(2) $$\begin{array}{c} y=\;\frac{x-\min\left(x\right)}{\max\left(x\right)-\min\left(x\right)}. \end{array}$$

### 2.2. Cubic Spline Interpolation

In the operation data set of a steel blast furnace from May to August, the detection time and frequency of each data variable are quite different. For example, the detection time interval of control variables such as gas permeability and oxygen-enriched flow rate is 1 hour, while the hot metal and slag are about 1.33 hours. In order to predict the hot metal silicon content normally, polynomial fitting, Gauss curve fitting, and cubic spline interpolation fitting methods are introduced to reduce the dimension of different control parameters [24]. Taking the oxygen enrichment rate as an example, 24 detection values per day are substituted into the three fitting functions as input samples to obtain the fitting function and curve, which reflect the changing trend of the oxygen enrichment rate in a day. By smoothing the curve, the fitting data of the oxygen enrichment rate at each moment can be obtained. According to the sampling time of the silicon content of the hot metal, 18 points on the curve are selected as the output, as is shown in Figure 2.

RETRACTED

Gauss curve and polynomial fitting focus on describing the overall trend of oxygen enrichment but do not require the curve to pass through sample points [25]. It can be seen from the comparison of the effect of the fitting algorithm in Figure 2 that the cubic spline interpolation method can better reflect the periodic changes of the oxygen enrichment rate in a day when the sample points are few. Therefore, in this paper, the cubic spline interpolation method is used to supplement and integrate the data, that is, curve fitting is carried out for a limited number of sample points. The corresponding value of *Y*-axis of the curve is obtained at a smaller time interval, which is used as the data set for the subsequent prediction of hot metal silicon content.

### 2.3. Analysis of Data Delay Based on the Combination of Spearman and Weighted Moving Average

Due to the large time lag of the blast furnace ironmaking process, it is difficult to accurately obtain the influence of control parameters such as the amount of coal injection and air pressure at different periods on the hot metal silicon content [26, 27]. Spearman correlation coefficient analysis is an algorithm for judging the degree of data association, and its value range is [−1, 1]. The larger the absolute value of the coefficient, the higher the correlation between the two attributes. Spearman correlation analysis is used to analyze the time series of different control parameters and silicon content in molten iron, which could better reflect the real-time change of blast furnace sample data. The formula for calculating Spearman's correlation coefficient is

(3) $$\begin{array}{c} \rho =\frac{\sum_{i=1}^{n}\left(x_{i}-\bar{x}\right)\left(y_{i}-\bar{y}\right)}{\sqrt{\sum_{i=1}^{n}{\left(x_{i}-\bar{x}\right)}^{2}\sum_{i=1}^{n}{\left(y_{i}-\bar{y}\right)}^{2}}}, \end{array}$$

where *x*_*i*_ is the control parameter of the *i*th; *y*_*i*_ is the silicon content of the *i*th furnace; and $\bar{x}$ and $\bar{y}$ are the average values of the control parameters and the silicon content of the hot metal, respectively.

Figure 3 shows the correlation analysis between some control parameters and hot metal silicon content under different time delays. It can be seen that the amount of coal injection and air permeability have the greatest correlation with the hot metal silicon content under 0 time delay. The hot air temperature and furnace top temperature have the greatest correlation with the silicon content of the hot metal under 3 time delays. The cold air pressure has the greatest correlation with the hot metal silicon content under 4 time delays. In this way, the correlation coefficients of all control parameters and the silicon content of the hot metal are obtained.

RETRACTED

Table 1 shows the correlation coefficients of some control parameters and the hot metal silicon content under different lag furnaces. Then, the blast furnace sample set was analyzed through the combination of multiple time series and the Spearman analysis method, and the relationship data between multiple control parameters and the hot metal silicon content was fitted. As the influence of various control parameters on the silicon content of molten iron is continuous, to simulate the internal reaction conditions of the blast furnace as much as possible, this paper uses the weighted moving average method (WMA) to trim the data [28]. Suppose the control parameter is *x*_*i*_, then the weighted moving average formula (equation (4)) is

(4) $$\begin{array}{c} {\hat{x}}_{it}=\;\frac{w_{1}x_{it}+w_{2}x_{i\left(t-1\right)}+\ldots +w_{n}x_{i\left(t-n+1\right)}}{w_{1}+w_{2}+\ldots +w_{n}}, \end{array}$$

(5) $$\begin{array}{c} w_{i}=\;\frac{b_{i}}{\sum_{l=1}^{m}b_{l}}, \end{array}$$

where ${\hat{x}}_{it}$ is the weighted moving average of the control parameter *x*_*i*_ at time *t*, *x*_*it*_ is the true value of the control parameter at time *t*, *b*_*i*_ is the Spearman correlation coefficient under time delay *i*, and *w*_*n*_ is the *n*th weight (the value of *n* need to be determined according to Spearman correlation coefficient).

As shown in Table 1, the Spearman correlation coefficients of multiple control parameters and different time delays are counted. Taking furnace roof temperature as an example, the absolute values of the Spearman correlation coefficients of furnace roof temperature are sorted in order, and the optimal furnace roof temperature threshold value 0.0632 is obtained through multiple experiments. That is, 0∼2 time delay furnace top temperature data are selected as the weight of the weighted moving average method. In the same way, set a reasonable threshold based on the principle of the number of weights being 3 and calculate the weights of other control parameters. Then it is substituted into formula (4) to obtain the prediction data set of molten iron silicon content based on time lag analysis.

RETRACTED

### 2.4. Backpropagation Neural Network

Backpropagation neural network (BPNN) is a multilayer feedforward network [29], and its structure is shown in Figure 4. Here, *x*_1_, *x*_2_, *x*_3_,…, *x*_*n*_ are the input values of *n* blast furnace control parameters, *y*_1_, *y*_2_, *y*_3_,…, *y*_*m*_ are *m* input values of the hot metal silicon content. *ω*_*ij*_ and *ω*_*kj*_ are the hidden layer and output layer weight, *θ*_*i*_ and *α*_*k*_ are the hidden layer and output layer thresholds, respectively. Its node element characteristic (transfer function) is Sigmoid type [30].

The BPNN updates the parameters through the generalized perceptron, and the adjustment of its weight and threshold formula are expressed as follows:

(6) $$\begin{array}{c} \text{total error criterion function: }E=\;\frac{1}{2}\overset{P}{\underset{p=1}{\sum }}\overset{L}{\underset{k=1}{\sum }}{\left(T_{k}^{P}-O_{k}^{P}\right)}^{2},\\ \text{output layer weight: }\Delta \omega_{ki}\;=\;\beta \overset{P}{\underset{p=1}{\sum }}\overset{L}{\underset{k=1}{\sum }}\left(T_{k}^{P}-O_{k}^{P}\right)\overset{`}{\varphi }\left({\text{net}}_{k}\right)y_{i},\\ \text{output layer thershold: }\Delta \alpha_{k}=\;\beta \overset{P}{\underset{p=1}{\sum }}\overset{L}{\underset{k=1}{\sum }}\left(T_{k}^{P}-O_{k}^{P}\right)\overset{`}{\varphi }\left({\text{net}}_{k}\right),\\ \text{hidden layer weight: }\Delta \omega_{ij}=\;\beta \overset{P}{\underset{p=1}{\sum }}\overset{L}{\underset{k=1}{\sum }}\left(T_{k}^{P}-O_{k}^{P}\right)\overset{`}{\varphi }\left({\text{net}}_{k}\right)\omega_{ki}\overset{`}{\emptyset }\left({\text{net}}_{k}\right)x_{j},\\ \text{hidden layer thershold: }\Delta \theta_{i}=\;\beta \overset{P}{\underset{p=1}{\sum }}\overset{L}{\underset{k=1}{\sum }}\left(T_{k}^{P}-O_{k}^{P}\right)\overset{`}{\varphi }\left({\text{net}}_{k}\right)\omega_{ki}\overset{`}{\emptyset }\left({\text{net}}_{k}\right). \end{array}$$

### 2.5. Genetic Algorithm

As the BPNN algorithm uses the gradient descent method to modify the weights and thresholds, it has an insufficient accumulation of the experience and has certain defects. These defects are specifically manifested as follows:

1. The learning efficiency is low and the convergence speed is slow
2. It is easy to fall into a local minimum state

To solve the above problems, genetic algorithm (GA) is introduced to optimize the parameters, to improve the convergence speed and achieve global optimization [31, 32]. The basic steps of the GA are as follows:

(1) Determine the real number code according to the number of weights and thresholds of the BPNN, and randomly generate the initial population.
(2) In order to achieve the global optimization of neural network training errors. The absolute value of the BPNN predictive error is taken as the fitness *F*, and the encoded individuals are transformed into decision variables in the problem space. The fitness function is as follows:
  (7) $$\begin{array}{c} F=k\left(\sum_{i=1}^{m}abs\left(y_{i}-{\hat{y}}_{i}\right)\right). \end{array}$$
Here, *y*_*i*_ and ${\hat{y}}_{i}$ are the true and predicted values of the silicon content of the *i*th hot metal, respectively, and *k* is the coefficient.
(3) Using the roulette method, according to the size of individual fitness, *p*_*i*_ probability selects some individuals with greater fitness from the population to form a mating pool. The formulas are as follows:
  (8) $$\begin{array}{c} f_{i}=\frac{k}{F_{i}}, \end{array}$$
  (9) $$\begin{array}{c} p_{i}=\;\frac{f_{i}}{\sum_{j=1}^{N}f_{i}}, \end{array}$$
where *N* is the number of populations, *F*_*i*_ is the fitness of the *i*th individual, and *k* is the coefficient.
(4) Use crossover and mutation operations to update the mating pool. The crossover operation uses the real number crossover method. The formulas are as follows:
  (10) $$\begin{array}{c} a_{ki}=a_{ki}1-b+a_{li}b, \end{array}$$
  (11) $$\begin{array}{c} a_{li}=a_{li}1-b+a_{ki}b. \end{array}$$
where *b* is a random number in the interval [0, 1].
(5) Repeat steps (2)–(4) until the convergence judgment is satisfied.

In summary, the GA-BPNN model is constructed. The flowchart is shown in Figure 5.

RETRACTED

### 2.6. Model Prediction and Error Analysis

Based on the traditional BPNN prediction model, the genetic algorithm is used to optimize the parameters to obtain the preliminary predictive results of the hot metal silicon content. However, the BPNN model optimized by genetic algorithm has a large error for the hot metal silicon content. The error analysis is shown in Figure 6. It can be seen that the error curve is almost the same as the changing trend of the hot metal silicon content, so it is inferred that the formation of the error is related to time series of the hot metal silicon content. In order to further improve the prediction accuracy, the autocorrelation analysis is carried out on the time series of the hot metal silicon content. The autocorrelation coefficient is used as the weight, the actual value of nearly 3 furnaces is input, the initial prediction error is the output, and the error analysis model is established. The predictive function of error analysis is also implemented by the GA-BPNN algorithm (details not included here). The training set and the test set are divided to optimize the parameters of the error prediction model. When the prediction accuracy becomes stable, the error prediction value is added to the preliminary prediction value of the silicon content of the molten iron in the next batch to obtain the revised prediction value of the hot metal silicon content. In summary, the Si-content in GA-BPNN hot metal error correction prediction model based on data optimization is shown in Figure 7.

RETRACTED

## 3. Result Analysis

### 3.1. Preliminary Prediction of the Model

To eliminate the dimension of each group of data, denoising and normalization processing are carried out for the selected predictive sample of hot metal silicon content. The cubic spline interpolation fitting model is used to realize the data integration of multiple detection periods. Spearman analysis and the weighted moving average method are combined to analyze the time lag of the integrated data, to obtain new data sets corresponding to control parameters and hot metal silicon content. The BPNN improved by genetic algorithm is used to predict. Select 1500 preprocessed blast furnace samples, of which 1000 are used as the training set and 500 are used as testing sets for model training. Due to a large amount of data in the training set, it is not conducive to model tuning, so the cross-validation method is used to train the model. Set the parameter *k* = 20, that is, divide the training sets into 20 parts. Then make preliminary predictions respectively, which can be expressed by the following formula:

(12) $$\begin{array}{c} \text{train}X=\left[{\left[x_{1}\right]}_{j},{\left[x_{2}\right]}_{j},{\left[x_{3}\right]}_{j},\ldots ,{\left[x_{39}\right]}_{j}\right]\;j=1∼50,51∼100,\ldots ,950∼1000. \end{array}$$

Here, train*X* represents the control parameter set used for training (all four-step prediction).

(13) $$\begin{array}{c} \text{train}Y_{i}={\left[S_{i}\right]}_{j+i-1}\;j=1∼50,51∼100,\ldots ,950∼1000. \end{array}$$

Here, train*Y*_*i*_ represents the training set label used for the *i*th prediction.

(14) $$\begin{array}{c} \text{test}X=\left[{\left[x_{1}\right]}_{j},{\left[x_{2}\right]}_{j},{\left[x_{3}\right]}_{j},\ldots ,{\left[x_{39}\right]}_{j}\right]\;j=1001∼1500. \end{array}$$

Here, test*Y*_*i*_ represents the control parameter set used for the test (all four-step prediction).

(15) $$\begin{array}{c} \text{test}Y_{i}={\left[S_{i}\right]}_{j+i-1}\;j=1001∼1500. \end{array}$$

Here, test*Y*_*i*_ represents the test set label used for the *i*th prediction.

Figure 8 shows the comparison between the preliminary predictive results and the actual value of 400 furnaces. It can be seen that the improved BPNN model based on genetic algorithm has basically realized the prediction of the hot metal silicon content, but the accuracy still needs to be improved.

RETRACTED

### 3.2. Error Analysis

Analyze the time series of the hot metal silicon content and obtain the autocorrelation coefficient of silicon content as is shown in Figure 9. The *X*-axis represents the number of furnaces, and the *Y*-axis represents the autocorrelation coefficient of silicon content. It can be seen that the furnaces with the greatest correlation with *n* furnaces are *n* − 1, *n* − 2, and *n* − 3 furnaces, and they show a decreasing trend. As is shown in Table 2, set the threshold to 0.2 and select the first *n* − 1, *n* − 2, and *n* − 3 furnace data as input for error reprediction. The error prediction is obtained (Figure 10). The genetic algorithm BPNN model is corrected through error analysis to obtain the corrected prediction value and compare it with the direct preliminary prediction result of the BPNN.

### 3.3. Model Evaluation

The predicted value of the error is added to the preliminary prediction result of the silicon content of the molten iron to obtain the revised predicted value of the silicon content of the molten iron. The comparison of the prediction results before and after the correction is shown in Figure 11. It can be seen that the predicted value corrected by error analysis is much closer to the real value. In order to quantitatively analyze the changes in prediction accuracy before and after correction, three evaluation indicators are introduced to analyze the model errors. They are root mean square error (RMSE), average absolute error (MAE), and average absolute percentage error (MAPE). It can be seen from Table 3 that the GA-BPNN model proposed in this paper is significantly smaller than the ordinary BPNN model in all three prediction errors, and the GA-BPNN model based on error correction achieves the best prediction effect.

## 4. Conclusion

The prediction of the hot metal silicon content plays a vital role in the temperature control and normal operation of the blast furnace. The methods of combining cubic spline interpolation fitting, Spearman analysis, and weighted moving average method are respectively proposed to optimize data. Based on the BP neural network model, genetic algorithm is used to optimize the parameters to improve the convergence speed of the model and achieve global optimization. Combined with autocorrelation analysis of hot metal silicon content, a correction model for the prediction of hot metal silicon content based on error analysis is proposed to further improve the accuracy of the prediction model.

The results show that the average absolute error of the prediction model for the correction of hot metal silicon content based on the data optimization is 0.05009, which has greatly improved the prediction accuracy compared to before the error correction.

RETRACTED

The model fully taps the value of limited data sets and has strong portability. In the subsequent development, the prediction accuracy of the model can be further improved through the 2-step and 3-step error analysis.

## Figures and Tables

**Figure 1:** Boxplot of hot metal silicon content.

**Figure 2:** Comparison and analysis of different curve fitting methods: (a) Gauss curve fitting, (b) quartic polynomial fitting, and (c) cubic spline interpolation fitting.

**Figure 3:** Correlation analysis of partial control parameters and hot metal silicon content at different time delays.

**Figure 4:** BPNN model.

**Figure 5:** GA-BPNN model.

**Figure 6:** The prediction error is compared with the real value.

**Figure 7:** Error correction prediction model of Si-content in GA-BPNN hot metal based on data optimization.

**Figure 8:** Comparison between the preliminary prediction results and the real value of hot metal silicon content.

**Figure 9:** Autocorrelation coefficient of hot metal silicon content.

**Figure 10:** Contrast of the actual error with the predicted error.

**Figure 11:** Comparison of prediction results before and after correction.

**Table 1:** The correlation coefficient between control parameters and hot metal silicon content.

Time delays	Coal injection	Air permeability	Hot air temperature	Cold air pressure	Furnace top temperature	Oxygen-enriched flow	Hot metal sulfur content
0	−0.3484	0.65588	−0.1251	0.3501	−0.0632	−0.1287	−0.2107
1	−0.0877	0.24513	0.1040	0.0780	−0.1153	−0.1840	−0.0021
2	0.0958	0.0149	0.2270	−0.2314	−0.2457	−0.1833	0.0013
3	0.1160	0.01286	0.2133	−0.3711	−0.0325	−0.0489	−0.0017
4	0.0033	0.22088	0.1224	−0.2829	−0.0317	0.0126	0.0009
5	−0.1350	−0.2999	0.0344	−0.0886	−0.0170	0.0172	−0.0026

**Table 2:** Error analysis of model data.

Error	*n* furnaces predictive value	*n* − 1 furnaces predictive value	*n* − 2 furnaces predictive value	*n* − 3 furnaces predictive value
−0.20534	0.40466	0.54235	0.4808	0.45264
0.09759	0.49759	0.40466	0.54235	0.4808
−0.00365	0.45635	0.49759	0.40466	0.54235
−0.23829	0.42171	0.45635	0.49759	0.40466
−0.00701	0.43299	0.42171	0.45635	0.49759
0.14438	0.47438	0.43299	0.42171	0.45635
0.2079	0.5279	0.47438	0.43299	0.42171
0.13273	0.44273	0.5279	0.47438	0.43299

**Table 3:** Error comparison analysis.

	RMSE	MAE	MAPE
BPNN	0.20182	0.16063	0.37609
GA-BPNN	0.18010	0.13549	0.27235
Corrected GA-BPNN	0.06749	0.05009	0.10474

## Data Availability

The data used to support the findings of this study are available from the corresponding author upon request.
